RETRACTED

# Factors affecting the green investment and assessing sustainable performance of firms in China

**DOI:** 10.1371/journal.pone.0296099

**Published:** 2023-12-21

**Authors:** Yufei An, Ghulam Rasool Madni

**Affiliations:** 1 School of Economics, Management and Law, Shaanxi University of Technology, Hanzhong, China; 2 Department of Economics, Division of Management and Administrative Science, University of Education, Lahore, Pakistan; Universiti Malaysia Kelantan, MALAYSIA

## Abstract

In the process of development, global economies are prioritizing environmental protection and firms are also recognizing the importance of minimizing environmental impact during production along with maximization of profits through green investments. It is vivid that green investments are vital for environmental preservation. So this paper contributes to literature by investigating the role of internal and external factors affecting the decision making of Chinese firms regarding adoption of green investments and impact of green investments on environmental, social, and economic performance of firms. The data is collected from directors/senior managers of the firms. We received 463 valid responses from listed companies with Shenzhen, Beijing, and Shanghai Stock Exchange. The “structural equation modeling” with “maximum likelihood estimation” is employed for empirical analysis. The empirical findings reveal that adaptation to climate change and its mitigation is the most important driver of green investment. Moreover, green investment positively contributes to enhancing the social, economic, and environmental performances of Chinese firms. Based on the findings of the study, green investment should be adopted as a corporate strategy by firms for profit maximization, competitive advantage, and improvement in social well-being without compromising the environment. Policy makers can promote green investment by offering policy instruments such as tax incentives, guaranteed credits, grants, and investor education. Training courses may be offered to raise environmental awareness among firms and the general public.

## 1. Introduction

The rapid development of China has resulted in significant costs on the environment. According to the “environmental performance index report” 2018, China stands at 120^th^ position out of 180 countries. Additionally, “more than 70% of large and medium-sized cities of China are not according to the air quality standards set by WHO” [1]. As a global economic player, China is now actively addressing environmental issues, including global warming. To this end, China has begun to align its domestic investment goals with the requirements of the green economy. Furthermore, China is an active member and supporter of the “Paris Climate Change Agreement”.

RETRACTED

There are numerous factors affecting the global environment while industrial activities are the main reasons for environmental deterioration. According to Zhang et al. [2], industrial activities of firms are widely believed to be the main cause of environmental problems. In fact, the emissions of SO, NO, and smoke from these activities are responsible for 88.15, 67.60, and 83.65 percent of total emission, respectively. Shen et al. [3] support this argument and found that 80% of environmental pollution is due to operations and production activities of firms in China. Despite this, Chinese firms have generally failed to invest in green initiatives due to the negative externalities of pollution [2,4]. Liao et al. [5] warn that prioritizing short-term economic growth over environmental concerns can have severe consequences. As public attention towards environmental issues grows, companies are under increasing pressure [6]. However, addressing environmental problems is not an overnight task for enterprises, and there are two main reasons limiting its progress. First, companies have to make additional investments that could hinder short run profit maximization objectives. Secondly, strong externalities of environmental pollution can affect the effectiveness of governance related to the environment if other enterprises do not participate. To meet environmental governance standards, firms must adopt sustainable development practices and revise their investment strategies [7].

Environmental degradation often leads to increased government regulations and stricter environmental standards. Firms may choose to invest in green initiatives to comply with these regulations and avoid penalties, fines, or legal liabilities. According to surveys, there are multiple factors that impact a firm’s decision to invest in green initiatives. One study by Cortez et al. [8] found that external determinants like environmental regulations, have an influence on a company’s green investments and financial performance. Li et al. [9] demonstrated that both external and internal factors guide companies towards investing in pollution reduction goals. Yu and Zhang [10] are of the view that external factors can also impact innovation and result in additional costs on manufacturing. Environmental regulations are the primary concern of previous literature investigating its role on technological innovation. However, other crucial factors, including green investments, have not received adequate attention. It has been demonstrated through empirical evidence from Korean and Chinese firms that financial performance and competitiveness can be improved through active environmental management [11]. Green investment is a promising strategy for environmental preservation, promotion of technological innovations, and effectively fulfilling a firm’s social responsibilities [12]. Green investments are beneficial for companies in several ways, as pointed out by previous studies. Firstly, they can serve as a signal of the company’s commitment to fulfilling social responsibilities, which can enhance corporate valuation [13]. Secondly, Li et al. [9] indicated that firms investing in green technology can access subsidies by the government, generate higher profits, and promote green marketing. The government of China is exploring recently how to encourage green investments among enterprises to support green development. For instance, green investments have gained popularity in the BRI project and there is remarkable increase in investment in renewable resources to achieve sustainable goals [14].

RETRACTED

Green investment options for Chinese firms can help promote sustainability and environmental responsibility while also potentially expanding their profits. Some promising avenues include investment in renewable energy like solar and wind power projects to operate the plants, which not only contribute to reducing the nation’s carbon footprint but also tap into the growing demand for clean energy sources [15–19]. Additionally, energy efficiency technologies, green building construction, and sustainable agriculture are other promising sectors for investment, offering opportunities to reduce resource consumption and greenhouse gas emissions. Furthermore, firms can produce environmentally friendly and recyclable products with environmental technology startups to foster sustainable growth [20]. With China’s commitment to ecological stewardship, embracing these green investments not only makes environmental sense but can also yield long-term financial benefits.

On the other hand, green investments can have a significant impact on the environmental, social, and economic performance of firms in various ways. Green investments in renewable energy and emission reduction projects can directly reduce a firm’s carbon emissions [4]. This not only contributes to combat climate change but can also lead to operational cost savings through energy efficiency. Moreover, investment in green technologies and research can lead to innovations and the development of environmentally friendly products and services [9]. The social impact of green investment occurs in the form of creation of employment opportunities, thus contributing to social development and poverty reduction [11]. Firms involved in green projects often engage with local communities, addressing their concerns and fostering positive relationships [13]. Moreover, reducing pollution and improving environmental conditions through green investments can lead to improved public health, reducing healthcare costs and increasing overall well-being [12]. Firms that embrace green investments can enhance their reputation and competitiveness, appealing to environmentally conscious consumers and investors. This can lead to increased market share and revenue having a great economic impact [14]. Investments in energy efficiency, waste reduction, and sustainable practices can result in cost savings over the long term, improving a firm’s financial performance. Moreover, green-focused companies may have better access to green finance opportunities, such as green bonds or loans with favorable terms, which can support their growth and development [15–18].

RETRACTED

To determine the factors affecting the green investment by Chinese firms has much significance in the literature of environmental preservation to save the environment and its implications for sustainable performance of firms. For a comprehensive understanding of factors affecting decisions of green investment by firms, more detailed and systematic evidence is necessary. In this study, comprehensive and novel evidence is provided regarding external and internal factors influencing the decisions of Chinese firms to engage in green investments. There is hardly any study exploring the factors affecting the decision making of Chinese forms for green investment and impact of green investment on environmental, social, and economic performance of Chinese firms. We empirically examined the influential factors of green investment using data obtained from 463 listed companies in the Beijing, Shanghai, and Shenzhen Stock Exchanges. The main objectives of the study are to examine the factors affecting the decision making of Chinese firms regarding green investment and impact of green investment on environmental, social and economic performance of the firms. This study contributes to the literature through many ways. Although there is extensive literature on green investment, there is limited literature examining the factors influencing Chinese firms’ decision-making for green investment at the micro-level. The firms are major contributors to environmental degradation so understanding the behavior for green investment is necessary for upgradation of industry and regional development. Understanding the factors that influence the decision making of firms for green investment is crucial for formation of effective policies to save the environment and resource efficiency. However, current evidence on the drivers of green investments is insufficient. The empirical results of the study depict that external and internal drivers have a positive and significant role for green investment. Moreover, green investments enhance the environmental, social and economic performance of the Chinese firms.

RETRACTED

After the introduction, section two describes the earlier literature and hypotheses of the study. Section three explains the materials and methods while section four highlights the estimated empirical results. Next section five discusses the estimated results and the last section concludes the paper.

## 2. Earlier literature and hypothesis

Green investment refers to the utilization of green capital and investment in provisions of environmentally friendly products, and activities aimed at preventing, mitigating, or compensating for environmental damage, like adopting energy-saving measures or transitioning to renewable energy sources [21]. There are several ways to define green investment. The OECD, for example, considers green investment as a broader concept that “is closely related to other investment approaches such as socially responsible investing (investing in line with social responsibility), ESG (environmental, social and governance) investing (investing in line with environmental, social and governance factors), sustainable, long-term investing, or similar concepts” [22]. Eyraud et al. [23] perceives green investments as “investment necessary to reduce greenhouse gas and air pollutant emissions, without significantly reducing the production and consumption of non-energy goods.” The key components of green investments are focused on reducing emissions from energy sources, including nuclear power, biofuels, and renewable energy. Moreover, in OECD [18] green investment report, “green investments refer to investments that are good for the environment, low carbon emissions and funded projects primarily in the field of renewable energy or clean tech companies, environmental technology or markets related to as clean, sustainable, and climate change investments.”

The study [19] tested the expanded model of Theory of Planned Behavior to find the factors affecting intentions of green investment in the Kingdom of Saudi Arabia. A questionnaire was sent to 550 graduates of agricultural and food sciences from public universities of the Kingdom. The PLS-SEM results showed strong positive effects of attitudes, knowledge of green investments, and commitment to green consumption on the intention of potential investors to make green investments. The findings did support a detrimental impact of subjective norms on the intention to make green investments. The findings also supported a moderating effect of religion on the associations between attitude and intention to make green investments.

RETRACTED

The study [20] evaluates the current situation of portfolio investment in carbon solution with a focus on emerging markets (EMs) using a dataset of 37000 mutual funds at global level. Investment funds related to green investments are primarily focused on the USA while China is far distant from the largest green fund investment. The allocation of green investments in EMs is hampered by a number of issues. In order to solve the multiple issues slowing down green investment in EMs, a comprehensive strategy is required. A greater knowledge is required about what steers green investment to some nations rather than others, and what fuels green investment in EMs.

Investments in renewable energy and green financing help to reduce climate change and accomplish sustainable development objectives. The study [21] used the theory of planned behavior (TPB) to evaluate the factors that affect households’ intention to invest in green projects. Through structured questionnaire interviews and random sampling, the primary data was gathered from Iranian households. It has been found through the use of structural equation modelling that attitudes, subjective norms, perceived behavioral control, evaluation of the regulatory framework, perceived risk, and perceived utility of power purchase agreements all have a significant impact on households’ intentions to invest in green projects. This study offers empirical results in addition to theoretical ideas that can help policymakers in the process of enabling families for green investment.

The primary factors influencing green investment are examined by the study [22]. Green credit lines, green private lending, and green bonds are the financial products that promote green investment. In this study, an illustration of giving green credit in exchange for changing a logistics company’s service delivery technology is provided. The institutional element, such as legislative and technical requirements for investment, has been discovered in addition to the financial factors influencing green investments. There is a conflict between the aim to boost foreign direct investment and technical standards and environmental laws. The term of budgetary financing utilization and its usefulness for promoting renewable electricity as a type of green investment project are defined in the discussion.

Since individual investors dominate the Chinese capital market, analyzing their green investing practices has both significant practical implications for successfully utilizing the green finance incentive mechanism as well as a relatively complete theoretical value [23]. The study first acquires and screens the motivating elements of individual investors’ green investment behavior based on literature research and a questionnaire survey. The impact of the herding effect, local preference, environmental awareness, media information, residential environmental pollution level, policy considerations, company image, and green investment desire on investment behavior were identified using logistic regression and other methods. Thirdly, the action courses of the driving elements are tested using a structural equation model, and six noteworthy influence paths are found among the eight factors.

RETRACTED

### 2.1. Internal drivers and green investment

Internal factors refer to factors that are specific to the investor and have a significant effect on their decision regarding green investment. For firms, internal drivers play a crucial role in their green investment decisions due to extensive energy consumption. These drivers include investing in innovative technologies, adopting environmental management systems, and displaying eco-labels [24]. To achieve sustainability, firms require internal and external efforts in association with strong coordination among various departments [25]. Financial performance and economic value are major factors that motivate firms to be environmentally responsible, such as reducing operational costs, increasing sales volume, and gaining market share [26]. Firms strive to be greener to secure competitive advantages among competitors and to create a positive image among customers. In Taiwan’s information and electronics industries, companies that invest more in green products have a great competitive edge [27]. The major internal drivers considered in this study are reputation of the firm, efficiency gains, financial performance, investor’s preferences, and organizational culture.

**H1.** Internal drivers positively and significantly affect the green investment decisions by Chinese firms.

### 2.2. External drivers and green investment

External factors refer to factors that are outside the control of the investor but have a significant influence on green investment decisions. External factors play a significant role in driving green investment decisions. These include increasing customer preference for environmentally responsible products and services, as well as the desire to minimize adverse environmental impacts [28]. As environmental awareness grows, the demand for green products is on the rise [29]. Firms are motivated to adopt green initiatives when there is supplier pressure, as suppliers prefer to do business with eco-friendly organizations [30]. Policy makers incentivize firms to adopt green technology through rewards such as tax breaks and lowered taxes [18]. Additionally, compliance with governmental and environmental regulations is a major factor that encourages firms to invest in green initiatives [31]. Therefore, external factors have a significant impact on green investment, and firms consider these factors when making green investment decisions [32,33]. The major external factors considered in this study are public financing, target market, incentives, regulations and legislation, climate change, consumers’ behavior, stakeholders’ behavior.

RETRACTED

**H2.** External drivers positively and significantly affect the green investment decisions by Chinese firms.

### 2.3. Environmental performance and green investment

Environmental performance is a firm’s capacity to decrease waste and emissions, hazardous substances, and environmental incidents [34]. To gain competitive advantages, businesses across various industries are now implementing strategic environmental performance programs [29]. Investment in green technologies, green innovations, and renewable energies improve the environmental performance. The earlier literature determined the relation between green investment and environmental performance. Chen and Ma [11] conducted an empirical study on Chinese firms and found that green investment has a positive effect on improving the environmental performance of a firm. Similarly, for the Indonesian manufacturing sector, Indriastuti and Chariri [32] found that green investment significantly enhanced sustainable performance. Ren et al. [33] further suggest that green investment is a vital driver for China’s sustainable development. They state that green investment negatively impacts environmental pollution by promoting energy conservation, emissions reduction, innovative technology development, and industrial infrastructure renovation [34]. Additionally, Asadi et al. [35] observed a positive impact of green investment on environmental performance of the Malaysian hotel industry. The hypothesis can be devised on the basis of above literature:

**H3.** Green investments by Chinese firms play a significant role to increase their environmental performance.

### 2.4. Economic performance and green investment

When referring to economic performance, improving the financial capacities due to adoption of green strategy are considered, which have allowed firms to surpass industry standards [36]. Green investment is considered a crucial factor in economic advancement, as green investment can positively affect organizational cost. Numerous studies [17,26,30,32] indicated that green investment significantly impacts economic performance. Asadi et al. [35] showed that green investment increases economic performance by reducing energy consumption, reducing waste treatments fees, and lowering penalty for environment related accidents. Additionally, Yannan et al. [36] are of the view that green investment enhances the sales of the manufacturing industry in China.

RETRACTED

**H4.** Green investments by Chinese firms play a significant role to maximize their economic performance.

### 2.5. Social performance and green investment

Organizations often prioritize economic objectives over other aspects, especially in the short term [36,37]. However, long run sustainability cannot be achieved by focusing solely on economic objectives [38]. To achieve sustainability in association with economic benefits, it is important to establish some criteria that may enhance social and environmental performance [39]. In addition to increasing employee satisfaction and retention, companies can benefit from addressing environmental concerns by improving community relations and enhancing their brand acceptance [7]. Furthermore, fostering social awareness among employees and attracting and retaining the right talent can yield various benefits [40]. According to Wagner [41], companies that prioritize social responsibility and accountability can attract top talent, retain customers, and foster innovations, contributing to social performance of firms. Yang [42] conducted a study exploring the relation between green investment and social livability in the Thai tourism industry, and found that green investment significantly improves social livability by creating employment opportunities for low-income individuals, generating "green" employment, reducing death rate, and improving social justice.

**H5.** Green investments by Chinese firms have a significant role in improvement of their social performance.

The Fig 1 highlights the conceptual framework of the study.

**Fig 1:** Conceptual framework.

## 3. Materials and methods

The study used an online questionnaire to gather data which was sent through emails and social media messengers. The survey questionnaire is placed in appendix. To develop the measurement tools, the researchers conducted a thorough analysis and review of previously published studies. The researchers developed six constructs and each of them with specific items. The sample was selected from companies listed on the Beijing, Shanghai, and Shenzhen Stock Exchanges. There are seven sections of the questionnaire; the first section is about general information about the company. The 2^nd^ and 3^rd^ parts examined the company’s internal and external factors affecting green investment decisions. The 4^th^ part evaluated the extent to which the companies implemented green investment in their operations. The 5^th^, 6^th^, and 7^th^ parts assessed the companies’ environmental, economic, and social performance, respectively. A five point Likert scale is used where 1 showing “strongly disagree” and 5 showing “strongly agree”. The survey questions were completed by executives, managers, or the most senior staff.

RETRACTED

The measures regarding green investment were derived from the work of Elzek et al. [43] and Chen and Ma [11] through six items, with one example being "The firm updates equipment-operating processes to save energy". The values of Cronbach’s α depict high internal consistency. The study [44] adopted and modified the internal and external factors affecting green investment. Each scale consisted of five items, with internal drivers including the “company’s culture towards environmental sustainability, and external drivers such as adaptation to/mitigation of climate change and ecological degradation”. The values of Cronbach’s α depict high internal consistency. The studies [45,46] developed the questionnaire items to measure environmental, economic, and social performance of firms. Examples of evaluating the influence of green investment on environmental performance include statements such as "Green investment helps reduce the impact of climate change and ecological degradation." The economic performance of firms is assessed using the statement "Green investment increases the company’s sales volume and profit margin". The social performance of firms is evaluated through the statement "Green investment enhances the quality of life". All values of Cronbach’s alpha show a high level of internal consistency. Initially, a pilot survey was conducted with 32 participants to assess the clarity, consistency, simplicity, and lack of ambiguity of the questionnaire. Upon receiving the feedback, some statements in the questionnaire were modified.

This research explores the factors affecting Chinese firms’ green investments and examines the extent to which such investments impact their environmental, economic, and social performance. A random sample of listed firms is selected, and an online questionnaire was administered to the senior officials of each company. The study’s purpose was clearly communicated, and participation was voluntary. Of the 650 questionnaires distributed, 463 were considered for statistical analysis. The time period of data collection was about three months (October-December 2022). The sample of 463 is sufficient for “structural equation modeling” (SEM) analysis, as it followed Nunnally’s [46] recommendation that “the sample size should be based on the number of items to be analyzed, with a case-to-item ratio of 10:1 being acceptable.” Additionally, 100–150 samples are required for “maximum likelihood estimation” [47,48] and Boomsma [49] suggests a sample of at least 200 for SEM.

RETRACTED

The collected data was analyzed using various statistical measures such as percentages, frequencies, means, and standard deviations. The validity and reliability are evaluated through “confirmatory factor analysis” (CFA) and “Cronbach’s alpha”. Convergence validity was established through the use of “average variance extracted” (AVE) and “composite reliability” (CR), and discriminant validity was determined using the “Fornell-Larcker criterion”. To determine “common method variance” (CMV), the “Harman single-factor test” is applied. Lastly, “structural equation modeling” (SEM) with “maximum likelihood estimation” (MLE) was utilized to test the hypotheses and establishment of mutual relationship among variables and their constructs.

## 4. Results

The demographic characteristics of the participants of the study are given in the following Table 1.

**Table 1:** Demographic characteristics.

Characteristics	No.	Percentage
Gender		
Male	418	90.3
Female	45	9.7
Age		
30 to less than 40 years	177	38.4
40–50 years	245	52.6
More than 50 years	41	9
Education		
University Degree	242	52.4
Master’s Degree	150	32.5
Doctoral Degree	70	15.1
Designation		
General Manager	322	69.55
Environmental Manager	108	23.33
Other	33	7.12
No. of Years at Current Position		
Less than 5 years	61	13.17
5–10 years	251	54.21
11–15 years	102	22.03
More than 15 years	49	10.58

On the basis of 463 valid responses, the study found that 90.3% of the participants were male while only 9.7% were female. Regarding age distribution, the majority of participants fell into the higher category, with ages ranging from 30 to less than 40 years (38.4%), followed by those between 40 and 50 years old (52.6%). The 9% participants were older than 50 years. In terms of educational qualifications, 52.4% of participants held a university degree, while 32.5% have a master degree and 15.1% have doctorate degree.

Table 2 depicts the descriptive statistics and the corresponding items. The participants reported high levels of commitment to green technology and energy conservation, encouraging eco-labeled goods and services, and upgradation of equipment to save energy, with mean scores ranging from 3.96 to 4.51. Internal drivers of green investment were rated higher by participants, with mean scores ranging from 4.21 to 4.92. Financial performance, specifically returns on green investments, was identified as the highest internal driver motivating management to adopt green investment. Participants strongly perceived external factors as significant predictors of green investments, with average mean scores ranging from 4.01–4.59. “Adaptation to/mitigation of climate change and adapting to continuous market changes” are the highest perceived external drivers affecting the decisions regarding green investment. Regarding the perceived impact of green investment on social, economic and environmental performance of firms, findings showed that participants believed that green investments reduce GHG emissions (environmental), increase the volume of sales of firms and their profit level (economic), and improve quality of life (social).

RETRACTED

**Table 2:** Descriptive statistics.

Construct	Item	Mean	SD	Factor Loading	Cronbach’s α	CR	AVE
Green Investment	1	4.13	0.88	0.812*	0.924	0.916	0.731
	2	4.01	0.84	0.741*			
	3	4.28	0.90	0.836*			
	4	4.36	0.83	0.827*			
	5	3.96	0.87	0.892*			
	6	4.51	0.92	0.823*			
External Drivers	7	4.02	0.93	0.863*	0.892	0.967	0.764
	8	4.26	0.82	0.819*			
	9	4.33	0.15	0.792*			
	10	4.59	0.82	0.826*			
	11	4.01	0.63	0.853*			
Internal Drivers	12	4.53	0.92	0.916*	0.913	0.893	0.772
	13	4.28	0.86	0.829*			
	14	4.92	0.87	0.873*			
	15	4.83	0.83	0.814*			
	16	4.21	0.79	0.846*			
Economic Performance	17	4.51	0.88	0.889*	0.881	0.893	0.779
	18	4.38	0.82	0.849*			
	19	4.29	0.83	0.871*			
Environmental Performance	20	4.39	0.82	0.923*	0.911	0.952	0.810
	21	4.85	0.80	0.917*			
	22	4.52	0.83	0.893*			
Social Performance	23	4.36	0.81	0.856*	0.900	0.823	0.871
	24	4.57	0.87	0.861*			
	25	4.26	0.82	0.937*			
RMR = 0.063 RMSEA = 0.079 CFI = 0.933 GFI = 0.917 RFI = 0.951 NFI = 0.902 IFI = 0.935 Normed chi square (x^2^ / df) = 2.993 p ˂ 0.001							

Note: * shows significance at 1%. RMR = Root mean square residual; IFI = Incremental fit index; RMSEA = Root mean square error of Approximation; CFI = Comparative fit index; GFI = Goodness of fit index; RFI = Relative fit index; NFI = Normed fit index.

The validity and reliability of constructs is determined through a CFA using MLE. Firstly, reliability of constructs was examined using CR and Cronbach’s α. The values of Cronbach’s α and CR are higher than 0.80 (threshold value), showing good internal reliability [48]. Secondly, discriminant and convergent validity is determined. For convergent validity, it is required that factor loadings should be at least 0.50 and coefficients of AVE should be at least 0.50 [50]. The results indicated that all items had factor loading over 0.50, and the coefficients of AVE exceeded 0.50, indicating good convergent validity. Various goodness of fit indices are utilized to determine the model’s fitness. The (x2/df) ratio was below 5, and the RMR score was 0.063, while the RMSEA score was 0.079, both below the acceptable threshold of 0.08. Additionally, the GFI, CFI, RFI, NFI, and IFI values were all greater than the recommended values of 0.90 [48,51]. Therefore, according to these indicators, the data fitted the measurement model well.

RETRACTED

The criterion used to examine discriminant validity in this study was the Fornell-Larcker [50] criterion, which states that “a construct is considered to have discriminant validity if its square root is greater than its correlation with other constructs”. The results of the analysis are presented in Table 3, where the diagonal numbers show square root of AVE for each construct. Moreover, all the latent variables have AVE square roots that are higher than their correlation with other variable, thus indicating a good discriminant validity. To reduce the possibility of common method variance (CMV) bias due to the use of a web based questionnaire, three methods are applied: anonymity, confidentiality, and honesty [52]. To further detect any CMV, a commonly used test “Harman’s single-factor test” is applied and findings show that only 39.8% of variance could be responsible for a single factor, indicating that CMV is not a significant issue [53].

**Table 3:** A Fornell–Larcker method for discriminant validity.

	Green Investment	External Drivers	Internal Drivers	Economic Performance	Environmental Performance	Social Performance
Green Investment	0.885					
External Drivers	0.526*	0.847*				
Internal Drivers	0.468*	0.453*	0.851*			
Economic Performance	0.373*	0.462*	0.516*	0.869*		
Environmental Performance	0.285*	0.391*	0.428*	0.587*	0.847*	
Social Performance	0.314*	0.276*	0.362*	0.237*	0.428*	0.843*

Note: * shows significance at 1%.

SEM method is used to investigate the effect of potential variables on green investment and analyzing influence of green investment on social, economic, and environmental performance of firms. The findings are presented in Table 4.

**Table 4:** Structural parameter estimate.

Hypotheses	Standardized Path Coefficient	t-values	Result
IF → GI	0.423*	6.583	Yes
EF → GI	0.396*	7.293	Yes
GI → EP	0.499*	9.389	Yes
GI → ECP	0.516*	6.398	Yes
GI → SP	0.437*	4.887	Yes
x^2^/df = 2.989* NFI = 0.931 RMSEA = 0.071 CFI = 0.917 RFI = 0.910 GFI = 0.901 IFI = 0.924 RMR = 0.058			

Note: * shows significance at 1%. IF = Internal factors; EF = External factors; GI = Green investment; EP = Environmental Performance; SP = Social performance; ECP = Economic performance

The findings of SEM highlight that all estimated paths are positive and significant, and thus all hypothesis are supported.

## 5. Discussion

China has experienced substantial environmental degradation in the past thirty years due to its rapid industrialization and modernization [7]. Despite criticism of its contribution to global environmental degradation, China is currently promoting the development and utilization of eco-friendly technologies. This study investigates the key drivers that affect green investments made by Chinese firms and examines how such investments have their impact on environmental, economic, and social performance. The findings of SEM analysis suggest several significant results. Firstly, the results support the first hypothesis, indicating that internal drivers have a positive and significant impact on green investment. Specifically, financial returns on green investment, efficiency gains, and a firm’s organizational culture towards environmental sustainability were found to be significant predictors of green investment implementation. The earlier literature also found a strong relation between financial returns and green investment [9,12,54] and suggested that a company’s environmental management sensitivity significantly affects environmental sustainability implementation [24]. Additionally, Chitimiea et al. [45] found that factors such as securing competitive advantages and developing environmental reputation are predictors of green investment. The green investment decisions of firms are influenced by a range of internal factors [55]. These internal factors can shape a firm’s strategic approach to sustainability and environmental responsibility. The organization’s culture and values play a crucial role [56]. Companies with a strong commitment to sustainability and environmental responsibility are more likely to prioritize green investments. In addition, the attitudes and commitment of top management can greatly influence green investment decisions. When leaders are committed to sustainability, it often permeates throughout the organization [19]. It is also found that firms with strong research and development capabilities may be more inclined to invest in innovative green technologies and solutions [17]. Companies aiming to improve operational efficiency may invest in green initiatives to reduce energy consumption, waste, and resource use, which can lead to cost savings [31]. Employee attitudes and engagement can also affect green investment decisions. A workforce that is environmentally conscious and supportive of sustainability goals can drive internal initiatives. It’s important to note that internal factors are interconnected, and their relative importance can vary from one company to another [12]. It is also found that external factors positively affect green investment. Therefore, for firms to implement green investment successfully, they should consider external factors like adapting to/mitigating climate changes, adopting the changing markets, and meeting the expectations of consumers and stakeholders regarding environmental sustainability. These findings align with previous research that has shown that adapting to climate change, market changes, meeting environmental expectations, and complying with government regulations are significant predictors of green investment implementation [11,22,44,54,57]. Green investment of firms in China, like those in other countries, are influenced by a variety of external factors like regulatory, economic, social, and technological factors. Government policies play a significant role in shaping green investment decisions. Policies that promote environmental protection, sustainability, and renewable energy can incentivize firms to invest in green projects [21]. For example, subsidies, tax incentives, and carbon trading schemes can make green investments more financially attractive. Stringent environmental regulations and standards can require firms to invest in green technologies and practices to avoid penalties and maintain their operations [18]. Moreover, the cost of green technologies and practices relative to traditional ones can influence investment decisions. As green technologies become more cost-effective, firms are more likely to invest in them.

RETRACTED

Consumer and market demand for environmentally friendly products and services can drive firms to invest in green initiatives [17]. Meeting these demands can lead to competitive advantages and increased market share. Public perception and reputation management are vital for businesses. Firms may invest in green initiatives to enhance their image and reputation, especially if they face public pressure to do so [25]. The specific impact of these factors can vary depending on the industry, company size, and the firm’s strategic goals. However, the overall trend in China, as in many parts of the world, is toward increased investment in green and sustainable practices due to growing environmental awareness and regulatory pressures.

It is revealed that green investment improves firms’ environmental performance. Therefore, investing in green practices and innovative technologies can lead to reduced greenhouse gas emissions, fewer environmental accidents, mitigation of environmental degradation, and improved environmental performance. Earlier literature also suggests that green investment is effective in mobilization of green capital, which can be used to offer environmentally friendly products, preserve natural biodiversity, and mitigate the adverse effects of climate change and environmental degradation [55]. Additionally, these findings align with the findings of Chen and Ma [11] who concluded that green investment promotes environmental performance of Chinese firms. Further, these findings are also in line with the data obtained from listed companies of China which highlighted that green investments help to boost environmental performance of Chinese firms and reduce environmental violation [18]. In the context of Indonesian firms, the findings of this study are supported by arguing that green investments positively and significantly have an impact on sustainable performance of firms. Yan et al. [54] collected the data of 3706 firms of 20 countries covering the time span of 2002–2013 and found a positive and significant relation between environmental performance and green investment. Therefore, it can be concluded that green investment enhances the environmental performance of firms.

RETRACTED

It is also found that green investment has a positive impact on the economic performance of firms. Specifically, it contributes to increasing sales volumes, profit margin, and market share, while also reducing long-term costs such as energy and water consumption. These results are consistent with previous research such as Chariri et al. [30], highlighting the positive correlation between financial performance and green investment in Indonesian companies. Similarly, other studies [11,17,30,32,35] have also highlighted that green investment is a major factor improving the economic performance of a firm, leading to reduced costs, increased value of firm, enhanced reputation, and a competitive advantage. The study [32] explained that “green investment may have an inverted U-shaped impact on economic performance, indicating a cutoff value beyond which further increases in green investment could negatively affect financial performance”. This could be due to companies losing focus on other product quality aspects when investing too much in green activities, which might result in an inability to offer better products to customers.

Lastly, the study shows a positive relation between green investment and firms’ social performance, suggesting that higher levels of green investment correspond to better social performance. These findings align with Abou-Liela’s [55] who found that green investment improves the quality of social life, like increased public welfare, higher satisfaction, and enhanced environmental awareness. Yang [42] also found a positive relationship between green investment on social livability in Thailand, which showed that green investment promotes social livability by creating "green jobs," promoting social justice.

RETRACTED

## 6. Conclusion

One of the prime objectives of this study is to determine the drivers influencing green investment by Chinese firms and how such investment has an influence on social, economic and environmental performance of firms. An online questionnaire is used to collect responses from senior officials of Chinese firms. We received 463 valid responses and data is analyzed using SEM. The findings indicate that both external and internal drivers significantly influence green investment, with climate change adaptation as the most prominent driver. Furthermore, green investment improves the social, economic and environmental performance of firms. Moreover, green investment is a source to promote sustainable performance.

This study has several theoretical implications derived from the findings of the study. Firstly, this study is an addition in the literature of green investment by providing a comprehensive understanding regarding the role of internal and external drivers influencing green investments, confirming its role in promoting sustainable performance and supporting the importance of aligning with stakeholders’ expectations. Although external drivers have higher impact on green investment as compared with internal drivers but both have positive and significant impact. Adaptation to climate change is the most influential factor of green investment. Secondly, it is found that green investment plays a pivotal role to enhance the sustainable performance of firms. The derived results revealed that green investment positively and significantly affects the economic, social and environmental performance of the firms. Thirdly, the legitimacy theory is also supported by the findings of the study which explains that public support can be gained through adopting such activities and practices which are according to expectations of the public and stakeholders [46], including the practices relevant to green investment. According to legitimacy theory, the findings of the study highlight that firms may gain their legitimacy from the public through caring about green investments mitigating the environmental degradation, greenhouse gas emissions and improving the living standard of the community. Additionally, it offers practical implications for organizations seeking legitimacy and public support. Fourth, there is hardly any study that examines the effect of internal and external factors on green investment in the context of Chinese firms, providing valuable insights for future research in other specific industrial sectors. Fifth, a theoretical framework is developed to determine the factors of green investments and its consequences on firms. The findings of the study are significant revealing the importance of this study for future research in other sectors.

RETRACTED

The study’s results offer several practical implications. Firstly, firms should consider both internal and external drivers when formulating strategic plans, especially in the context of environmental preservation, as well as considering the financial returns of green investment. Secondly, investment in green technology such as renewable energy, and eco-label products can enhance the social, economic and environmental performance of a firm so their competitive advantage may be sustained. So firms may make investments in green innovations to enlarge their profits and save the environment. It will enhance the economic, social and environmental performance of Chinese firms. Thirdly, green investment can be used as a corporate strategy for profit maximization while protecting the environment. Fourth, authorities should play a leading role regarding promotion of green investments through development of policies having the objective to promote green investment. Policy makers can also promote green investment by offering policy instruments such as tax incentives, guaranteed credits, grants, and investor education. Fourthly, awareness about the environment can be raised through training courses. Fifthly, green investments enhance the quality of life, boost employment opportunities, and foster a relationship with the community. Sixthly, firms should pay serious attention to raise the environmental awareness among their employees through training courses regarding the significance of green investments.

There are also some limitations of this study. The study is conducted on a randomly selected sample of Chinese firms to determine the factors influencing and outcomes of green investments, which may limit the generalization of its findings to other countries. Future research could involve a larger and more diverse sample for more comprehensive insights. The study treated the effect of internal and external factors on green investment as a uni-dimensional construct comprising five factors. Future research could consider examining the influence of each driver individually on green investment, as well as exploring additional variables. Thirdly, the study relied on an online questionnaire completed by the participants based on their subjective perspectives. To provide a deeper understanding of the phenomenon, mixed-method approaches involving quantitative and qualitative data collection methods could be used in future research.

## Supporting information

S1 File https://drive.google.com/file/d/1YtTQmmUwbfnPkOgmh-lany6S3Mi3fAYl/view?usp=sharing.
(PDF)

S1 Data https://docs.google.com/spreadsheets/d/12LvgRQ6AnpB-OhMYji76q5XxWmdIpyf5/edit?usp=drive_link&ouid=104935469773789258540&rtpof=true&sd=true
(XLSX)

RETRACTED

## References

[1] World Health Organization. World health statistics 2016: monitoring health for the SDGs, sustainable development goals. 2016. https://apps.who.int/iris/handle/10665/206498

[2] ZhangG.; GaoY.; LiJ.; et al. China’s environmental policy intensity for 1978–2019. Sci Data. 2022, 9, 75. doi: 10.1038/s41597-022-01183-y 35277526 PMC8917127

[3] ShenW.T.; YuX.; ZhongS.B.; GeH.R. Population Health Effects of Air Pollution: fresh Evidence from China Health and Retirement Longitudinal Survey. Front Public Health. 2021, 23(9), 779552. doi: 10.3389/fpubh.2021.779552 35004584 PMC8733201

[4] ZhengS.; KahnM.E. A New Era of Pollution Progress in Urban China? The Journal of Economic Perspectives. 2017, 31(1), 71–92.

[5] LiaoL.; DuM.; ChenZ. Air pollution, health care use and medical costs: Evidence from China. Energy Econ. 2021, 95, 105132.

[6] AlamM.S.; MuhammadA.; ChuC.C.; UgurS. Does corporate R&D investment affect firm environmental performance? Evidence from G-6 countries. Energy Econ. 2019, 78, 401–411.

[7] SharifA.; GodilD.I.; XuB.; SinhaA.; RehmanS.A.; JermsittiparsertK. Revisiting the role of tourism and globalization in environmental degradation in China: fresh insights from the quantile ARDL approach. J Clean Prod. 2020, 272, 122906.

[8] CortezM.C.; AndradeN.; SilvaF. The environmental and financial performance of green energy investments: European evidence. Ecol. Econ. 2022, 197, 107427.

[9] LiX.; DuK.; OuyangX.; LiuL. Does more stringent environmental regulation induce firms’ innovation? Evidence from the 11th Five-year plan in China. Energy Econ. 2022, 112, 106110.

[10] YuY.; ZhangN. Environmental regulation and innovation: Evidence from China. Glob. Environ. Chang. 2022, 76, 102587.

[11] ChenY.; MaY. Does green investment improve energy firm performance? Energy Policy. 2021, 153, 112252.

[12] IraldoF.; TestaF.; FreyM. Is an environmental management system able to influence environmental and competitive performance? The case of the eco-management and audit scheme (EMAS) in the European union. J. Clean. Prod. 2009, 17, 1444–1452.

[13] MartinP.R.; MoserD.V. Managers’ green investment disclosures and investors’ reaction. J. Account. Econ. 2016, 61, 239–254.

[14] FanQ.; LiuJ.; ZhangT.; LiuH. An Evaluation of the Efficiency of China’s green investment in the “Belt and Road” countries. Struct. Chang. Econ. Dyn. 2022, 60, 496–511.

[15] UN-ESCAP. Economic and Social Survey of Asia and the Pacific 2010: Year-end Update. United Nations Building Rajadamnern Nok Avenue Bangkok 10200, Thailand. 2010.

RETRACTED

[16] OECD. Green Growth and Developing Countries. A Summary for Policy Makers. 2012.

[17] AliedanM.M.; AlyahyaM.A.; ElshaerI.A.; SobaihA.E.E. Who Is Going Green? Determinants of Green Investment Intention in the Saudi Food Industry. Agriculture. 2023, 13, 1047.

[18] OECD. Towards Orderly Green Transition: Investment Requirements and Managing Risks to Capital Flows. 2023. https://www.oecd.org/investment/investment-policy/towards-orderly-greentransition.pdf

[19] RahmaniA.; MashayekhJ.; AboojafariR.; NaeiniA.B. Determinants of households’ intention for investment in renewable energy projects. Renewable Energy. 2023, 205, 823–837.

[20] VarnaliiZ.S.; CheberyakoO.V.; MiedviedkovaN.S.; BorysenkoO.A.; NikytenkoD.V.; KaletnykO.V. Economic and Business Management. 2023. CRC Press.

[21] LiC.; ZhangY.; HouG.; MaM. Analysis of Driving Factors and Action Path of Green Investment Behavior of Individual Investors. Highlights in Business, Economics and Management. 2023, 9, 33–43.

[22] MadniG. R. Meditation for role of productive capacities and green investment on ecological footprint in BRI countries. Environmental Science and Pollution Research. 2023, 30(28), 72308–72318. doi: 10.1007/s11356-023-27478-0 37170048

[23] EyraudL.; ZhangC.; WaneA.A.; ClementsB.J. Who’s Going Green and Why? Trends and Determinants of Green Investment. IMF Working Papers. 2011, 296.

[24] AbdouA.H.; HassanT.H.; DiefE.; MoustafaM. A description of green hotel practices and their role in achieving sustainable development. Sustainability. 2020, 12, 9624.

[25] KrausS.; BurtscherJ.; VallasterC.; AngererM. Sustainable Entrepreneurship Orientation: A Reflection on Status-Quo Research on Factors Facilitating Responsible Managerial Practices. Sustainability 2018, 10, 444.

[26] PaulA.K.; BhattacharyyaD.K.; AnandS. Green Initiatives for Business Sustainability and Value Creation (Advances in Business Strategy and Competitive Advantage (ABSCA), 1st ed.; IGI Global: Hershey, PA, USA, 2017.

[27] ChenY.; LaiS.; WenC. The influence of green innovation performance on corporate advantage in Taiwan. J. Bus. Ethics. 2006, 67, 331–339.

[28] BhuiyanM.A.; KahouliB.; HamaguchiY.; ZhangQ. The role of green energy deployment and economic growth in carbon dioxide emissions: evidence from the Chinese economy. Environ Sci Pollut Res. 2023, 30, 13162–13173.10.1007/s11356-022-23026-4PMC948579436125680

[29] TaoT.; MadniG.R.; YasinI. Mediating the performance of social organizations in context of social and organizational innovations in China. PLoS ONE. 2023, 18(3): e0281720. doi: 10.1371/journal.pone.0281720 36961796 PMC10038268

[30] ChaririA.; NasirM.; JanuartiI.; DaljonoD. Determinants and consequences of environmental investment: An empirical study of Indonesian firms. J. Asia Bus. Stud. 2019, 13, 433–449.

RETRACTED

[31] CuiH.; WangR.; WangH. An evolutionary analysis of green finance sustainability based on multi-agent game. J Clean Prod. 2020, 269, 121799.

[32] IndriastutiM.; ChaririA. The role of green investment and corporate social responsibility investment on sustainable performance. Cogent Bus. Manag. 2021, 8, 1960120.

[33] RenS.; HaoY.;WuH. How Does Green Investment Affect Environmental Pollution? Evidence from China. Env. Resour. Econ. 2022, 81, 25–51.

[34] PengZ.; MadniG.R.; AnwarM.A.; YasinI. Imperative of Institutions for Effective Relationship Between Economic Performance and Ethnic Diversity. Journal of the Knowledge Economy. 2023. 10.1007/s13132-023-01195-y

[35] AsadiS.; PourhashemiS.O.; NilashiM.; AbdullahR.; SamadS.; YadegaridehkordiE.; et al. Investigating influence of green innovation on sustainability performance: A case on Malaysian hotel industry. J. Clean. Prod. 2020, 258, 120860.

[36] YannanD.; AhmedA.A.A.; KuoT.; MalikH.A.; NassaniA.A.; HaffarM.; et al. Impact of CSR, innovation, and green investment on sales growth: New evidence from manufacturing industries of China and Saudi Arabia. Ekon. Istraživanja. 2022, 35, 4537–4556.

[37] XieS.; MadniG.R. Impact of Social Media on Young Generation’s Green Consumption Behavior through Subjective Norms and Perceived Green Value. Sustainability, 2023, 15, 3739.

[38] HassanT.H.; SalemA.E.; AbdelmoatyM.A. Impact of Rural Tourism Development on Residents Satisfaction with the Local Environment, Socio-Economy and Quality of Life in Al Ahsa Region, Saudi Arabia. Int. J. Environ. Res. Public Health. 2022, 19, 4410. doi: 10.3390/ijerph19074410 35410089 PMC8998635

[39] ShabirM.; AliM.; HashmiS.H.; BakhshS. Heterogeneous effects of economic policy uncertainty and foreign direct investment on environmental quality: cross-country evidence. Environm Sci Pollut Res. 2022, 29,2737–2752. doi: 10.1007/s11356-021-15715-3 34378130

[40] UllahF.; JiangP.; ElamerA.A.; OwusuA. Environmental performance and corporate innovation in China: the moderating impact of firm ownership. Technol Forecast Soc Chang. 2022,184,121990.

[41] WagnerM. ‘Green’ Human Resource Benefits: Do they Matter as Determinants of Environmental Management System Implementation? J. Bus. Ethics. 2013, 114, 443–456.

[42] YangX. How Does Green Investment Influence on Tourism Development in Thailand? J. Environ. Manag. Tour. 2022, 13, 1047–1058.

[43] ElzekY.S.; GaafarH.A.; AbdelsamieH. Evaluation of Sustainable Tourism Investment in Tourism Businesses: Evidence from Egypt. J. Fac. Tour. Hotel. -Univ. Sadat City 2020, 4, 42–58.

RETRACTED

[44] QianC.; MadniG.R. Encirclement of Natural Resources, Green Investment, and Economic Complexity for Mitigation of Ecological Footprints in BRI Countries. Sustainability. 2022, 14, 15269.

[45] ChitimieaA.; MinciuM.; MantaA.; CiocoiuC.N.; VeithC. The Drivers of Green Investment: A Bibliometric and Systematic Review. Sustainability. 2021, 13, 3507.

[46] NunnallyJ.C.; Psychometric Theory 3E. Tata McGraw-Hill Education: New York, NY, USA, 1994.

[47] HairJ.F.; BlackW.C.; BabinB.J.; AndersonR.E. Multivariate Data Analysis: Pearson New International Edition; 2014. Pearson Education Ltd, Essex, UK.

[48] ZhaoJ.; MadniG.R. The impact of economic and political reforms on environmental performance in developing countries. PLoS ONE, 202, 16(10), e0257631. doi: 10.1371/journal.pone.0257631 34610016 PMC8491874

[49] BoomsmaA. The Robustness of Lisrel against Small Sample Sizes in Factor Analysis Models. 1982. North-Holland Publ. Co., Amsterdam, The Netherlands.

[50] FornellC.; LarckerD.F. Structural Equation Models with Unobservable Variables and Measurement Error: Algebra and Statistics. J. Mark. Res. 1981, 18, 382.

[51] NancarrowC.; BraceI.; WrightL.T. Tell me Lies, Tell me Sweet Little Lies: Dealing with Socially Desirable Responses in Market Research. Mark Rev. 2001, 2, 55–69.

[52] PodsakoffP.M.; MacKenzieS.B.; LeeJ.; PodsakoffN.P. Common method biases in behavioral research: A critical review of the literature and recommended remedies. J. Appl. Psychol. 2003, 88, 879. doi: 10.1037/0021-9010.88.5.879 14516251

[53] TranT.T.T.; DoH.N.; VuT.H.; DoN.N.M. The factors affecting green investment for sustainable development. Decis. Sci. Lett. 2020, 9, 365–386.

[54] YanS.; AlmandozJ.; FerraroF. The Impact of Logic (In)Compatibility: Green Investing, State Policy, and Corporate Environmental Performance. Adm. Sci. Q. 2021, 66, 903–944.

[55] Abou-LielaM.M. Green Investment of Heritage Environments a Doorway to a Life of Quality. In Proceedings of the 1st International Conference on Towards a Better Quality of Life, Technische Universität Berlin Campus El Gouna, El Gouna, Egypt, 4–26 November 2017.

[56] ZhangZ.; MadniG.R.; NaeemJ. Unleashing the horizons of labor quality, digitalization on upgradation of industrial structure in Asian economies. PLoS ONE. 2023, 18(7), e0288866. doi: 10.1371/journal.pone.0288866 37463163 PMC10353783

[57] ShuwangZ.; MadniG.R.; YasinI. Exploring the Mutual Nexus of Social Capital, Social Innovations and Organizational Performance. Sustainability. 2022, 14, 11858.

